# Tetramethylpyrazine Improves Monocrotaline-Induced Pulmonary Hypertension through the ROS/iNOS/PKG-1 Axis

**DOI:** 10.1155/2022/1890892

**Published:** 2022-03-24

**Authors:** Dong-Peng Yang, Wen-Peng Dong, Yong-Chao Yang, Yuan-Yuan Zeng, Ying Liu, Zhu Dong, Xi-Miao Ma, Yi-Qiu Cao, Yi-Zhou Bai, Bo Yang, Xiao-Wu Wang

**Affiliations:** ^1^The First School of Clinical Medicine, Southern Medical University, Guangzhou, China; ^2^Department of Cardiovascular Surgery, Guangzhou Red Cross Hospital, Jinan University, Guangzhou, China; ^3^Department of Cardiovascular Surgery, People's Liberation Army General Hospital of Southern Theater Command, Guangzhou, China; ^4^Department of Cardiovascular Surgery, The First Affiliated Hospital of Anhui Medical University, Jixi Road 218, Shushan District, Hefei 230032, China; ^5^Guangdong Cardiovascular Institute, WHO Collaborating Center for Research and Training in Cardiovascular Diseases, Guangdong Provincial People's Hospital, Guangdong Academy of Medical Sciences, Guangzhou 510080, China; ^6^Guangzhou University of Chinese Medicine, Guangzhou 510010, China; ^7^Jiangmen Wuyi Hospital of TCM, Jiangmen, Guangdong 529000, China; ^8^Department of Cardiovascular Surgery, Zhujiang Hospital, Southern Medical University, Guangzhou 510280, China

## Abstract

**Background:**

Tetramethylpyrazine (TMP), a potent anti-free radical and anti-inflammations substance, has been demonstrated to possess a direct vessel relaxation property. This study aimed to evaluate the effect of TMP treatment in pulmonary hypertension (PH) and test the hypothesis that TMP prevents or reverses the process of PH.

**Methods:**

Rats (*n* = 36) injected with 50 mg/kg of monocrotaline (MCT) subcutaneously 4 weeks to develop PH were then randomized to TMP (5 mg/kg per day) for another 4 weeks. Hemodynamics was evaluated via the right ventricle. Pulmonary vessels structural remodeling and inflammation were examined by histologic and transmission electron microscopy observation. The expression of inducible nitric oxide synthase (iNOS) and cGMP-dependent protein kinases 1 (PKG-1) was detected by immunohistochemical staining and Western blot. Generation of reactive oxygen species (ROS) and antioxidation species was measured by biochemical analyses.

**Results:**

MCT increased PH and right ventricle hypertrophy. TMP alleviated pulmonary arterial pressure elevation, leukocyte infiltration, and structural remodeling of pulmonary arterials induced by MCT successfully. TMP treatment significantly increased the PKG-1 expression and suppressed the iNOS expression. The activity of superoxide dismutase (SOD), glutathione peroxidase (GSH), and catalase (CAT) was significantly higher than control group, while malondialdehyde (MDA) levels were lower compared with MCT group.

**Conclusion:**

TMP can suppress established MCT-induced PH through the ROS/iNOS/PKG axis. The underlying mechanisms may be associated with its anti-inflammatory, antioxidant, and antiproliferative properties in pulmonary arterial.

## 1. Introduction

Pulmonary hypertension (PH) is characterized by intimal lesions, medial hypertrophy, and adventitial thickening of precapillary pulmonary arterial. This is leading to a progressive increase in pulmonary vascular resistance [1]. The consequence of this increases right ventricle afterload, leading to right ventricle (RV) hypertrophy and ultimately heart failure and death. Demographics and epidemiology studies show an increased ratio of PH among older people [2, 3]. Most therapies for PH are designed to reduce pulmonary arterial resistance by inducing vasodilatation and to provide symptomatic relief, but the remodeling of vessels structure is still beyond control, and PH-related mortality remains unacceptably high. Current clinical practices starve for improvements in both conditions [4].

It is unlikely that one factor or gene mutation will explain all forms of PH, but it is well accepted that all subtypes of PH share a similar underlying pathology as well as a common hemodynamic diagnosis. Modern medicine touches its bottleneck on lots of diseases, such as to prevent the process of PH and traditional medicine shows a potent effect on it. Tetramethylpyrazine (TMP) (or TMP, 2, 3, 5, 6-TMP; TMP) is one of the alkaloids extracted from the rhizome of TMP Chuanxiong in 1957. This compound has been synthesized and used to treat several cardiovascular complications, including vascular diseases [5]. Direct relaxation of vessels by TMP has been indicated in vascular tissues and smooth muscle cells, exhibits effects on antioxidant, anti-inflammatory activities, modulates various inflammatory reactions, and has protective effects on multiple organs and systems [6, 7]. We hypothesis that TMP attenuates the PH process through its vasodilatation, antioxidant, anti-inflammatory, and antiproliferation properties.

To confirm our hypothesis, we choose a monocrotaline (MCT)-induced established rats PH model [8], which simulates the key pathology of human PH, including oxidative stress, leukocyte infiltration, vascular remodeling, and right ventricular hypertrophy. Our research is carried out particularly to test whether TMP exerts beneficial effects on oxidation, inflammation, and endothelia dysfunction in MCT-induced PH.

## 2. Methods

### 2.1. Animals

The animal use protocol was approved by Guangdong Medical Laboratory Animal Center ethics committee (Grant No.: 4400720007336). All animal care, breeding, and testing procedures were approved by the Laboratory Animal Users Committee at Guangzhou General Hospital of Guangzhou Military Command. Rats were housed in a temperature-, humidity-, and light-dark cycle-controlled environment with free access to food and water; all animals have 2 weeks to acclimatize the new environments.

### 2.2. Animal Models of PH

PH was generated in adult male Sprague–Dawley (SD) rats, weighing 250 g, by one subcutaneous injection of MCT (50 mg/kg; Sigma, St. Louis, MO, USA) or equal volume solvents (as control group). For the TMP efficacy study, rats developed into PH were randomized divided into MCT Group (MCT, *n* = 12) and TMP-treated Group (MCT+ 5 mg/kg TMP; *n* = 12) for an additional 4 weeks. Rats that were injected with solvents and receiving MCT act as the control group (*n* = 12).

### 2.3. Hemodynamic Measurement

4 weeks after TMP treatment, rats were anesthetized, incubated, and ventilated with a small animal ventilator (ALC-V8; ALCBIO, Shanghai, China) (500 mL/min·kg) in room air. Hearts were exposed via left thoracotomy. 24-F single use syringes with a fluid-filled catheter was inserted into the RV and left ventricle (LV) under direct vision to measure the pressure of RV and LV, respectively. The hearts and lungs were then harvested immediately, and the right ventricular and left heart (left ventricular plus septum) were weighed separately.

### 2.4. Transmission Electron Microscopy (TEM)

The hilum of the right lung was harvested and cut into pieces (1 mm × 1 mm × 1 mm) and fixed in electron microscopy of special glutaraldehyde (2.5%). Ultrathin sections were collected on 500-meshnickel grids, counter-stained with 5% uranyl acetate and lead citrate, and examined using a Hitachi H-7650 transmission electron microscope (Hitachi H-7650, Tokyo, Japan).

### 2.5. Histologic and Immunohistochemical Analyses

Lung tissue sections were prepared and stained with elastic a hematoxylin-eosin (H&E) stain. Morphometric analysis was performed on muscular arteries with the external diameter in the ranges of 50 to 99 *μ*m and 100 to 200 *μ*m. The medial wall thickness of each artery was calculated by the following formula:

(1) $$\begin{array}{c} \text{medial wall thickness}\left(\%\right)=\frac{\left(\text{cross}-\text{sectional area}\right)}{\left(\text{cross}-\text{sectional area}-\text{lumen area}\right)}\times 100\%. \end{array}$$

For each rat, 10 to 15 vessels were counted and the average value calculated.

The remaining tissue sections of the lung were subjected to immunostaining (GTVision III Shanghai Chain) with antibodies against induced nitric oxide synthase (iNOS) (ab205529, Abcam, Cambridge, UK) and cGMP-dependent protein kinase 1 (PKG-1) (ab90502, Abcam). The expression levels and activity of iNOS and PKG-1 were calculated as optical density observed by Image-Pro Plus application software.

### 2.6. Western Blotting

Proteins were extracted from the lung tissues that were frozen before to evaluate the effect of TMP on iNOS and PKG-1. Western blotting was performed by means of monoclonal antibodies to iNOS (ab205529, Abcam) and PKG-1(ab90502, Abcam). The proteins were detected as described in the instructions. Densitometric analysis was performed with (Image-Pro Plus) in each specimen.

### 2.7. Biochemical Analysis of Oxidative Stress

Lung tissues (100 ± 5 mg) were homogenized in a pre-cold mortar and pestle. Homogenates were then centrifuged at 4°C, 12000 g for 10 min (Micro 17R SN: 41519150). The ratio of reduced/oxidized glutathione (GSH/GSSG), malondialdehyde (MDA) content, as well as superoxide dismutase (SOD) and catalase (CAT) activity in lung tissues were determined as described in kit instructions. Kits used in testing were provided by Winching (Nanjing China).

### 2.8. Statistical Analysis

The statistical analysis was conducted using the Statistical Package for Social Science 23.0 (SPSS Inc, IL, USA). All data are given as the mean ± standard error (SEM). The analysis of variance between two groups was determined by one-way ANOVA. *P* < 0.05 was accepted as statistically significant.

## 3. Results

### 3.1. TMP Reversed the Process of MCT-Induced PH

PA medial wall thickness increased significantly after MCT treatment and TMP treatment significantly reversed the increase, i.e., suppressed the pulmonary vascular remodeling. MCT injection exacerbated the outlook of lungs and microstructure was indiscriminated with leukocyte infiltration (Figures 1(a) and 1(b)), and the changes were improved after TMP treatment (Figures 1(a)–1(c)). MCT injection increased the rats' body weight, but TMP treatment increased the body weight compared with the MCT group (Figure 1(b)). In addition, mean RV pressure (mRVP) was significantly elevated in rats challenged with MCT. TMP treatment significantly decreased the mRVP (Figure 1(c)). The RV hypertrophy was significantly increased in rats challenged with MCT and decreased after TMP treatment (Figure 1(d)).

### 3.2. MCT Treatment Seriously Affects the Ultrastructure of Pulmonary Artery

MCT treatment seriously affects the ultrastructure of pulmonary artery (Figure 2). ECs, SMCs, and membrane collagen fiber thickness were improved after TMP treatment (Figure 2). In the control group (control), the endothelial surface of the artery was regular, endothelial cells were distinctly (not shown). After MCT injection, shapes of SMC changed from spindle into irregular and surrounded with increased collagen fiber (Control-SMC, MCT-SMC, MCT-CF), endothelial cells attached loose to the basal lamina and the shape was changed into cubic or columnar and dropped into lumen (MCT-EC). TMP treatment improved this entire situation effective (MCT + TMP).

### 3.3. Suppressed iNOS and Enhanced PKG-1 Were Associated with Experimental PH

Immunohistochemical and Western blotting analyses (Figures 3(a)–3(c)) revealed that the expression of iNOS in the lung tissue was increased significantly in the MCT treatment groups compared with the control group, but the PKG-1 expression was significantly decreased. However, TMP treatment could reverse the expression of iNOS and PKG-1. These results declared that TMP could suppress iNOS expression and enhance PKG-1expression.

### 3.4. TMP Inhibited Oxidation Stress Induced by MCT

In MCT treatment groups, the levels of SOD, GSH, and CAT were significantly decreased while MDA was increased as compared to the control group (Figures 4(a)–4(d)). However, TMP treatment harvested a significant increase in SOD, GSH, and CAT activities yet decreased levels of MDA as compared with the MCT group (SOD (219.49 ± 3.11) vs. (166.19 ± 5.14), GSH (0.77 ± 0.03) vs. (0.51 ± 0.02), CAT (34.26 ± 0.98) vs. (25.91 ± 1.03), respectively. These results suggested that TMP treatment significantly improved oxidation stress induced by MCT.

## 4. Discussion

In our study, TMP significantly reduced the pulmonary artery pressure of MCT-P and, improved right ventricular hypertrophy and pulmonary artery muscularization. Transmission electron microscopy showed that TMP intervention inhibited MCT-PH endothelial cell necrosis and inhibited the proliferation and migration of pulmonary artery smooth muscle cells. Pulmonary artery wall connective tissue is reduced, pulmonary artery fibrosis is inhibited, and right ventricular hypertrophy is reduced. This is consistent with the previously reported results of TMP anti-inflammatory, inhibiting fibrosis and cell proliferation [7], indicating that TMP can act on pulmonary artery cells and the right ventricular myocardium and provides direct evidence for TMP to treat PH [5, 6]. TMP is cheap and has been widely used in the treatment of cardiovascular and cerebrovascular diseases. Its research on the prevention and treatment of PH has also been enriched, and it is expected to become an ideal drug for the treatment of PH.

Increased pulmonary artery pressure and right ventricular hypertrophy are the core pathological manifestations of PH, which are well reflected in MCT-PH. TMP can significantly reduce pulmonary artery pressure and reverse right ventricular hypertrophy to a certain extent. Pathological and ultrastructural observations confirmed that pulmonary artery smooth muscle hyperplasia and endothelial cell injury are particularly prominent in MCT-PH, which has important reference value for the pathological mechanism of PH in the acute stage. Further observation and research found that the expression of protein kinase PKG-1 related to pulmonary artery relaxation in MCT-PH lung tissue was significantly reduced, while the expression of iNOS increased. TMP has a particularly prominent regulatory effect on iNOS, and especially PKG-1.

iNOS is a kind of nitric oxide synthase (NOS) family of enzymes that can induce a large amount of NO produced by tissue inflammation. Studies have shown that iNOS and its induced product NO can regulate biological processes including glucose and lipid metabolism, nitro-oxidative stress, protein nitrification, cell damage, apoptosis, angiogenesis, cell proliferation, and migration. It plays an important role in the process of sepsis, asthma, rheumatoid arthritis, and other diseases, and it is the main mediator of vasodilation and hypotensive shock of septic [9–11]. In our study, TMP has a significant inhibitory effect on iNOS, which may be the molecular mechanism to prevent and treat PH. Seimetz et al. found that iNOS subcellular and cellular localization are important factors for its health and disease functions [12]. Through subcellular localization observation, we found that TMP can significantly reduce the expression of iNOS in granulocytes and smooth muscle cells and maintain its expression at a low level. This may be the molecular mechanism of TMP to maintain the pulmonary artery vasodilation function.

Inhibition of myosin light chain phosphorylation through the NO/cGMP/PKG pathway is a classic pathway for PKG to exert a vasodilator effect [13]. In our study, we found that the decrease of PKG-1 expression in the MCT-induced PH lung tissue and the increase of pulmonary artery pressure and right ventricular hypertrophy has a strong consistency. TMP can significantly increase the expression level of PKG-1, reduce pulmonary artery pressure, and improve right ventricular hypertrophy. Studies have shown that PKG-1 can improve pulmonary vascular remodeling, inhibit platelet activation and aggregation, and improve heart failure [14, 15]. The intervention of PKG-1 on biological processes includes increasing the uptake of glucose by cells, reducing mitochondrial oxidative stress, and inhibiting endothelial contraction induced by oxidative stress. PKG-1 can also inhibit TGF-*β*1, inhibit ERK phosphorylation, inhibit Rho A/Rho kinase activation, and other signal pathways to reduce pulmonary vasoconstriction, inhibit the proliferation of pulmonary vascular endothelial cells, and reduce pulmonary vascular remodeling [14, 16–18]. In addition, PKG-1 activates SMC-specific gene expression through the Elk-1-SRF signaling pathway to maintain its normal function [19]. It can also regulate cofilin activity to increase the tight junctions between cells, inhibit SMC migration, and inhibit small pulmonary artery muscularization, right ventricular hypertrophy, and achieve the effect of reducing pulmonary artery pressure [17, 18, 20]. This may be the molecular mechanism by which TMP regulates PKG-1 to prevent and treat PH.

Transmission electron microscopy results show that TMP significantly reduces the proliferation and migration of pulmonary artery smooth muscle cells, increases the tight junctions between cells, and improves the structural disorder of the pulmonary artery wall, which are the basis for the function of the pulmonary artery. MCT-induced PH pulmonary artery endothelial cells can see vacuoles, the membrane collapses and ruptures, and the organelles are exposed and edema, which is similar to pyrolysis. Endothelial cells may have many forms of death such as necrosis and pyrolysis. Pathological observation showed that there was granulocyte infiltration around the pulmonary artery. In our study, immunohistochemical protein subcellular localization shows that iNOS was mainly concentrated in granulocytes, and the expression of PKG-1 was relatively concentrated in the pulmonary artery. This phenomenon indicates that the effect of iNOS on PKG-1 is achieved mainly through the interaction between cells. Studies have shown that ROS can change the upstream and downstream factors of the cGMP-PKG signaling pathway [21, 22]. ROS induces the uncoupling of NO synthase (NOS), causing less NO and more nitrification products [22]. The oxidation of sGC reduces the response to NO. PKG-I*α* itself is also a target of ROS. On the other hand, PKG-1 promotes the phosphorylation of serine 116 on NOS, participates in the endogenous regulation of basic NOS3 activity, and can also directly inhibit the vasoconstrictor activated by ROS and exert cardiovascular protection [20, 22]. In this study, we found that TMP treatment reduced MDA levels and increased SOD, GSH, and CAT levels in MCT-induced PH. This was in agreement with the findings of Mohammadi et al. [23]. Their study confirmed that long-term administration of methylsulfonylmethane could attenuate MCT-induced PH in rats by modulating oxidative stress and antioxidants.

The therapeutic effect of TMP on PH has been verified in many other experimental PH [6, 24], but its mechanism still needs to be further sorted. Relevant studies have shown that TMP inhibits the production of iNOS in N9 microglia induced by lipopolysaccharide by blocking the MAPK and PI3K/Akt signaling pathways and inhibiting intracellular ROS [25]. It can also protect rat brain blood/reperfusion deficiency by inhibiting the expression of NADPH oxidase and iNOS [26]. TMP plays an important role in numerous ischemia, inflammation, and hyperplasia related studies, by inhibiting inflammation and oxidative stress, antiproliferation, improving tissues, and organ remodeling [6, 27]. Based on the long-term clinical application of TMP, good curative effect, low price, and good oral absorption, it is expected to become an ideal drug for the clinical treatment of PH. More clinical and basic research studies are expected.

## Figures and Tables

**Figure 1:** TMP reversed the process of MCT-induced PH. (a) Representative over view of lift lungs of rats and photomicrographs (magnification: 200×) of H&E-stained of lung sections. Monocrotaline-injection rats (MCT) (B) exhibit serious tissue damage, pulmonary vascular media hypertrophy, and mononuclear cell infiltration compared the control group. TMP-treated rats. (C) showed significant improvements of lung tissue, prevention of pulmonary vascular remodeling, and absorption of infiltration (MCT + TMP). (b) Limited body weight increasing was induced by MCT treated, this limitation was partly broken by TMP treatment. (c) Peak RV systolic pressure developed progressively in MCT-injected rats and TMP treatment prevented development of pulmonary hypertension. (d) Adaptive RV hypertrophy was demonstrated by RV weight: (LV + S) weight ratio in MCT-injection rats. MCT treatment prevented RV hypertrophy. *N* = 12 per group. Data were mean ± SD, ^##^*P* < 0.01 vs. control group. ^*∗∗*^*P* < 0.01 vs. MCT group. PH, pulmonary hypertension.

**Figure 2:** Transmission electron microscopic images. SMC = smooth muscle cell; CF = collagen fiber; EC = endothelial cell; EF = elastin fiber; L = lumen; SEL = subendothelial layer.

**Figure 3:** iNOS and PKG-1 expression in rat lungs. (a and b) iNOS and PKG-1 expression were measured by immunohistochemical analysis in three groups; there was a marked upregulation of iNOS (arrow in i-MCT) (a) and downregulation of PKG-1 (arrow in P-MCT) (b) in the lungs from MCT treated rats, downregulation iNOS and upregulation PKG-1after TMP treatment (arrow in i-MCT + TMP, P-MCT + TMP). (c) Western blot analysis demonstrated the iNOS and PKG-1 expression in rat lung homogenates. The bar graph showed iNOS and PKG-1 levels obtained from quantitative densitometry analysis. *N* = 12 per group. Data were mean ± SD, ^##^*P* < 0.01 vs. control group. ^*∗∗*^*P* < 0.01 vs. MCT group.

**Figure 4:** TMP inhibited oxidation stress induced by MCT. (a–d) Biochemical analysis in rat lung homogenates demonstrated increased lungs oxidative stress after MCT treatment. The levels of SOD (a), CAT (b), and GSH (c) significantly increased, while MDA content (d) decreased perspective in the TMP treatment group. *N* = 12 per group. Data were mean ± SD, ^##^*P* < 0.01 vs. control group. ^*∗∗*^*P* < 0.01 vs. MCT group. SOD, superoxide dismutase; GSH, glutathione; CAT, catalase; MDA, malondialdehyde.

## Data Availability

The data used to support the findings of this study are available from the corresponding author upon request.
